# A multi-layer neural network-based evaluation of MHD radiative heat transfer in Eyring–Powell fluid model

**DOI:** 10.1016/j.heliyon.2025.e41800

**Published:** 2025-01-16

**Authors:** Muflih Alhazmi, Zahoor Shah, Muhammad Asif Zahoor Raja, Nafisa A. Albasheir, Maryam Jawaid

**Affiliations:** a Department of Mathematics, College of Science, Northern Border University, Arar, Saudi Arabia; b Department of Mathematics, COMSATS University Islamabad, Islamabad Campus, Pakistan; c Future Technology Research Center, National Yunlin University of Science and Technology, 123 University Road, Section 3, Douliou, Yunlin, 64002, Taiwan, ROC; d Department of Mathematics, College of Sciences and Arts (Magardah), King Khalid University, Magardah, 61421, Saudi Arabia

**Keywords:** Artificial intelligence, Multi-layer, Neural network, Eyring-Powell fluid, Magnetic hydrodynamics, Bayesian regularization procedure

## Abstract

In the modern era, artificial intelligence (AI) has been applied as one of the transformative factors for scientific research in many fields that could provide new solutions to extremely complicated and complex physical models. In this paper, a multi-layer neural network combined with Bayesian regularization procedure (MNNs-BRP) is utilized to evaluate the model MHD radiative heat in non-uniform heating Eyring Powell fluid (EPF-MHD-RHS). The mixed convection parameter, Prandtl number, and heat emission or immersion parameter are studied in relation to momentum and heat transfer. To facilitate analysis, governing partial differential equations (PDEs) are converted into ordinary differential equations (ODEs) only with the aid of similarity transformations. From there, a dataset is created and later trained, tested, and validated by the MNNs-BRP model for efficient estimating of fluid models. The MNNs-BRP model is robust and demonstrates high accuracy, which compares well with the benchmark solutions. Performances of which are confirmed by metrics like error histograms, mean squared-error (MSE) check-ups, and regression analysis with MSEs all over the interval [10^−09^ – 10^−04^] to ensure a sustained model. The obtained outcomes indicate that the model built and implemented utilizing a neural network offers precise performance ranging from 3.25E-13 to 5.41E-13 with a mean error of around 3.25E-13, 1.56E-11, 5.41E-13, 2.97E-12, 1.03E-11, 2.05E-12, 1.49E-12, and 5.01E-12, across eight different circumstances, suggesting improved capability and reliability of the developed predictive model. After careful review and analysis, we have found that the temperature of the fluid decreases with the increase of Prandl number, while an inverse result is noticed with heat emission. However, the velocity of the fluid have an increasing trend with increasing values of mixed convection parameter, and heat generation or absorption parameter. In contrast the velocity profile have a decreasing trend with the increasing values of magnetic field parameter and stratification parameter. This work on integrating AI into this classical fluid dynamics problem is an entirely new paradigm that involves a smart combination of computational strategies with advanced physical modeling techniques. Our investigation is not just raising the bar for predicting complex fluid dynamics but also showing how AI can truly transform the entire research domain of fluid mechanics and related scientific disciplines. All the numerical and graphical illustrations attained by employing the AI-based techniques authenticates the solution methodology for the evaluation of fluid dynamics problems.

**Table:** Nomenclature

*u, v*	Components of fluid velocity	*c*_*p*_	Specific heat (fluid)
*μ*	Fluid's kinematic Viscosity	*g*	Gravitational acceleration
*ρ*	Fluid density	*k*	Thermal conductivity
*Q*	Heat generation/absorption	*q*_*r*_	Roose land approximation
*T*	Temperature	*σ∗*	Stephan Boltzmann constant
*K∗*	Absorption coefficient	*τ*_*w*_	Shear stress
*Re*_*x*_	Local Reynolds number	*M*	Magnetic field's influence
*σ*	Fluid's parameter	*ε*	Material parameter
*λ*	Mixed convection parameter	*γ*	Heat emission/immersion parameter
*e1*	Stratification parameter	*Nr*	Thermal radiation parameter
θ(η)	Fluid's temperature profile	*Pr*	Prandtl number
*PDEs*	Partial differential equations	$f^{\prime }\left(\eta \right)$	Fluid's velocity profile
*TPF*	Two-phase flow	*scn*	Scenario
*EPF-MHD-RHS*	MHD radiative heat in non-uniform heating Eyring Powell fluid	*ODEs*	Ordinary differential equations
*A∗*^*,*^*B∗*	Coefficient of heat absorption/generation effect	*Sce*	scenarios
Fig.	figure		
**AI Terms**			
BRP	Bayesian regularization procedure	AI	Artificial Intelligence
MNNs	multi-learning neural networks	Eh	Error Histogram
Sg	Solution Graph	MSE	Mean square error
Rg	Regression analysis	Pg	Performance curve graph
Ae	Absolute error	Ts	Training state
Ea	Error auto correlation	Ic	Input error cross correlation
TS	Time series		

## 1 Introduction

Newtonian magnetohydrodynamic (MHD) flows of non-Newtonian fluids have emerged as a significant area, with numerous applications in engineering and industrial processes. MHD effects are especially important in influencing the fluid flows of electrically conducting fluids — an enormously influential family that include metallic melts, heat transport and coolant channel systems for fusion reactors among many others. The broad theoretical foundation of MHD in terms of Maxwell's equations which lays the basis for understanding the interaction between field and flow, results in a relatively comprehensive method to model such systems [1]. Moreover, knowledge gained from studies of the solar wind and extended MHD turbulence [2] also help to understand fluid behavior in these systems which are important for both astrophysical as well as industrial applications. In particular, Gautam et al. analyze non-Newtonian MHD bioconvection flow of nanofluid due to nonlinear thermal radiation with a few heat sources/sinks, showing the substantial features and its influence on fluid motion as well as thermal fields. Further, Hameed and Nadeem on unsteady MHD flow over a porous plate have been recommended studying the influence of magnetic fields in extra to analyzing fluid motion via porous media [3,4]. As per Nguyen and Nguyen [5] the theme of this work is to investigate incompressible non-Newtonian fluid flow dynamics hence, it eases the understanding of modeling these fluids in different technological realms. Their combined work illuminates specific issues connected to the reliable prediction of fluid behavior in various cases and Irgens explores non-Newtonian flow rheology from basics, essential for research understanding processes being followed through elaborated explanations. His detailed review significantly clarifies what is going on with such fluids and how they might be used successfully in industrial settings [6] (see Fig. 1, Fig. A, Fig. G, A, and G).

**Fig. 1:** Geometry of the problem.

**Fig. A:** Graphic visualization of multi-layer neural networks.

From high-temperature environments thermal radiation is of equal importance when analyzing such fluid flows. Radiation affects not only thermal boundary layers but also the long-range heat transfer in applications (e.g. nuclear reactors, aerospace systems and energy conversion technologies). The complexity also increases when we consider environmental and chemical parameters affecting the behavior of Eyring-Powell fluids. Specifically, this analysis in complex settings has been expanded recently with some comparative studies. Hussain et al. an investigation has been considered of heat transfer and fluid flow past a convectively heated porous wedge ambitiously, the effects induced by chemical reaction are taken into account rein both steady (BVP). Furthermore unsteady (BVG), subjecting an Eyring-Powell Fluid formulation. Khan A. and Ali studies on the unsteady gyrotactic microorganisms sensing flow of variable thermal characters in Eyring-Powell nanofluids [7,8]. The influence of non-uniform heat sources or sinks is known to be extremely important in various systems when heating/cooling are not homogeneous across the system (e.g. different temperature gradients, local production of energy within a facility). Non-uniform heating which induces temperature gradients is common in processes used for e.g., drying technologies, cooling in electronic devices and manufacturing of composites. The work by Oke (2022) studied the non-linear shear stress interactions of a modified Eyring-Powell fluid flow and Jabeen focused on diffusion effects in stratified convective flows. Other research across various sub-disciplines has to do with boundary layer radiation, and non-uniform heating — important in a variety of engineering applications involving thermal management as well as cooling systems [[9], [10], [11], [12], [13], [14]]. Recent studies focused on the use of different models of fluid dynamics in order to study the properties of nanofluids under different physical and thermal conditions. Das et al. [15] discussed and analyzed the irreversibility of triply stratified bio Marangoni convection in external flow-influenced Powell Eyring nanofluid, incorporating the working of entropy generation. Shaw et al. [[16], [22]] studied 3D MHD convective Darcy-Forchheimer Casson hybrid nanofluid flows over a rotating disk with the Cattaneo-Christov heat flux, Joule heating, and radiation. Nonlinear thermal radiation has been considered, as has entropy analysis and thermal performance. Concomitantly, Sen et al. [17] examined entropy generation and heat and mass transfer features in hybrid nanoliquids flow under MHD and nonlinear radiation, enhancing the assessment of thermodynamic irreversibility. Shaw et al. [[18], [21]] studied hydromagnetic slip flow and thermal performance through magnetic power-law hybrid nanofluids by considering Hall and ion slip currents along with modified Fourier's law, especially in Maxwell fluids operating at low Prandtl numbers. Mohanty et al. [19] extended this examination to nonlinear radiative cross-ternary hybrid nanofluid movement over a stretching cylinder in view of its utilization in industry and reversible or irreversible thermodynamics. Shaw et al. [20] studied the hydrothermal-fluidic characteristics for Oldroyd B fluid with hybrid nanostructures supported by exploring low and moderate Prandtl numbers, furthering understanding of heat transfer and flow characteristics in GNFs. The majority of these works have in common with S. Shaw having insightful impacts towards the understanding of nanofluids, hybrid nanostructures, and an element of irreversibility in the assessment of fluid flow mechanisms under varied thermal and magnetic circumstances. Altogether, the present contribution helps in enhancing the knowledge regarding the hybrid nanofluid flow behaviors within a range of industrial and scientific applications.

Once a fluid flow over a stretching sheet — such problem is more interesting as well applicable to several industrial processes like polymer sheet manufacturing, glass blowing and metal extrusion. The boundary layer flow which is formed by the stretching of the sheet results in a velocity field that plays an important role on momentum and thermal transport inside fluid. As the electrically conducting fluid is subjected to a magnetic field perpendicular to the sheet, it behaves when undergoing interaction with such fields. Understanding these interactions is critical for developing effective thermal management systems in next-generation manufacturing. Recent research investigates various aspects of thermal and fluid dynamics. Studies have explored the impact of heat sources and magnetic fields on natural convection in concentric annuli, as well as the effects of Newtonian heating and cooling in permeable regions. Additional work examines temperature-dependent heat sources and MHD effects on transient convective flow, while further analysis addresses MHD interactions and radiative effects on non-Newtonian fluids over stretching sheets, including activation energy impacts [[23], [24], [25], [26], [27], [28]]. In recent studies, fluid dynamics phenomena are discussed with special emphasis on non-Newtonian fluids with reference to physical state and temperature. MHD two-phase flow and radiation of an incompressible read more ≫ viscoelastic UCM fluid through a porous space with slip boundary conditions was explored thermally by Zeb et al. [29]. In another study, Zeb et al. [30] used Lie group analysis to investigate the double diffusive MHD tangent hyperbolic fluid flow of a stretching sheet with extensive implications for heat and mass transfer. Zeb et al. [31] further extended the study for Carreau fluid with the impacts of Arrhenius activation energy and melting heat transfer for a stretching sheet for purposes of material processing. Ullah et al. [32] advanced this aspect by analyzing magnetohydrodynamic tangent hyperbolic fluid boundary layer flow over a stretching sheet. Further, using an analytical method, Ullah et al. [33] analyzed the effect of melting and activation energy for magnetized transient flow of Prandtl Eyring fluid, considering Cattaneo-Christov heat flux for enhancement of heat transfer. In combination, these works provide an overview of highly nontrivial flow dynamics and can be used as a basis for numerous practical applications in industries and technologies.

The Eyring-Powell fluid model has been chosen for this study due to its ability to represent non-Newtonian fluids with a more accurate non-linear relationship between shear stress and shear rate than conventional models like the power-law fluid. Recent investigations have delved into the dynamics of thermal and fluid systems under magnetic fields [34]. This article [35] has explored the time-dependent behavior of MHD thermal fluid flow in permeable cavities. Another research focuses on heat transfer involving nanomaterials and magnetic fields within enclosures, emphasizing the influence of MHD on thermal efficiency. This model is particularly effective in scenarios where fluids exhibit both shear-thinning and normal stress effects, which are crucial for accurate modeling in industries like cosmetics, biomedicine, and petrochemical processing. Analyzing the interplay between MHD, radiation, and non-uniform heat sources/sinks on a stretching sheet offers a clear understanding of their impact on momentum and thermal profiles. This research investigates how these combined factors affect Eyring-Powell fluids, aiming to enhance the efficiency of systems needing precise thermal and flow management, such as in cooling high-temperature devices and developing advanced materials. Many Researchers have carried out investigation in various aspects of non-Newtonian fluid dynamics, including the use of ternary nanoparticles to enhance heat transfer in MHD flows. They have also analyzed the effects of temperature- and concentration-dependent parameters on MHD behavior using numerical methods. Additionally, advancements include solutions for chemical reactions and viscous dissipation in non-Newtonian MHD flows with thermal radiation on nonuniform stretching sheets. Further investigations have examined the impact of thermal radiation on mixed flow over stretching sheets, providing comprehensive insights into heat and mass transfer phenomena [[36], [37], [38], [39], [40]].

In a recent time, several studies have focused on tackle challenging fluid mechanics problems with improved efficiency and effectiveness by employing artificial intelligence-based schemes. Researchers faced difficulties exploring different fluid problems like nonlinear problems and multidimensional problems with traditional numerical approaches. This landscape has changed due to the application of AI-based algorithms, neural networks, and machine learning schemes. A novel study [41] has utilized the application of neural networks to analyze the unsteady three-dimensional flow of Eyring-Powell magneto-nanofluids. Z. Shah [42] has employed the computational AI-based technique to study the dynamics of a contracting cylinder for the cross magneto-nanofluid flow model and for convective Eyring-Powell magneto-nanofluid dynamics [43]. In a recent study, researchers have designed neural networks with Bayesian distribution [44] and stochastic computing approaches [45] for analyzing and modeling various fluid behavior and interactions. The application of LBMA is demonstrated to variable viscosity models and electrically conducting fluids [46], novel Bayesian stochastic networks for Williamson fluids [47], and machine learning investigations into tri-magnetized Sutterby nanofluids with Joule heating [48]. Furthermore, recent articles have focused on Eyring-Powell nanofluids with Darcy-Forchheimer slip [49], thermal exchange in dissipative ternary nanofluids [50], bioconvective micropolar nanofluids [51], and tuberculosis with medicine immunity impact [52], with the application of AI-based procedures. All these advancements highlight the importance of artificial intelligence in fluid dynamics-related problems and provide novel ideas to deal with such intricate problems [[53], [54], [55], [56]].

The key contributions of the proposed computational methodology are listed below:

• The study uses an optimized multi-neural network model with Bayesian Regularization (MLNNs-BRP) for analysis of MHD radiative heat in non-uniform heating Eyring Powell fluid (EPF-MHD-RHS).
• The solution of non-linear partial differential equations (PDE) on EPF-MHD-RHS is suitably converted into a system of ODEs through the use of similarity transformations that makes more convenient analyses thereon.
• Using the Adam numerical method in an advanced environment called “Mathematica”, a full reference dataset for MLNNs-BRP is created. The model is built in such a way that crucial physical parameters are allowed to vary mixed convection parameter, Prandtl number, stratification parameter
• The comprehensive simulations are conducted on the proposed MLNNs-BRP, under different scenarios with the EPF-MHD-RHS in order to evaluate its accuracy and robustness. It is then compared against the reference dataset in order to validate its performance.
• The precision of the proposed MNNs-BRP validation is confirmed by utilizing error histogram, convergence of MSE, performance curve charts, and regression analysis.

This work is unique from prior studies since, for the first time, the utilization of a multi-layer neural network as an AI-based technique is proposed to model and analyze the pertinent MHD radiative heat transfer phenomenology of the Eyring-Powell fluid. This approach is superior to the numerical and analytical methods used in the past because it is a faster, more accurate, and more robust solution method. Moreover, the outcomes of magnetohydrodynamics, radiation, and the non-Newtonian characteristic of the Eyring-Powell fluid are incorporated for analysis, and essentially they have not been investigated by other previous researchers. The ability to predict and optimize such complex fluid behavior under various physical parameters using the application of neural networks is an important achievement. This study on MHD radiative heat transfer using the Eyring-Powell fluid model may be applied in the future to industrial and engineering processes like polymer production, chemical industries, and cooling systems in power plants, among others, since non-Newtonian fluids are widely used. The addition of magnetic fields and radiative heat effects takes on even more applicability in such applications as electromagnetic pumps, nuclear power plant cooling, or high-end space vehicle cooling systems. The originality of this work is in using a multi-layer neural network to model non-linear fluid dynamics, both stationary and time-dependent, with the incorporation of MHD forces and radiation effects in parallel with the conventional numerical and analytical approaches.

## 2 Problem description

Consider the two-dimensional flow of an incompressible EPFM over a stretching sheet that moves along x-axis with time at constant speed *U*_*w*_ = *ax*. The temperature of the fluid near the wall is *T*_*w*_ and far from it reaches at value *T*_*∞*_ with a free stream velocity for zero velocity bulk flow. In the energy equation, there is a factor of heat emission and absorption.

The stress tensor in the Eyring-Powell model is expressed as outlined by Powell and Eyring (1944) and further elaborated by Steffe (1996).

(1) $$T=\left\{\mu +\frac{1}{\beta \dot{\gamma }}\sinh^{-1}\left(\frac{1}{c}\dot{\gamma }\right)\right\}A_{1}\text{,}$$

where

(2) $$\dot{\dot{\gamma }=\sqrt{\frac{1}{2}tr{\left(A_{1}\right)}^{2}}}\text{,}$$

Consider the equations of continuity and momentum equation from Ref. [57]:

(3) $$\frac{\partial u}{\partial x}+\frac{\partial v}{\partial y}=0\text{,}$$

(4) $$u\frac{\partial u}{\partial x}+v\frac{\partial u}{\partial y}=\left(v+\frac{1}{\rho \beta c}\right)\frac{\partial^{2}u}{\partial y^{2}}-\frac{1}{2\rho \beta c^{3}}{\left(\frac{\partial u}{\partial y}\right)}^{2}\frac{\partial^{2}u}{\partial y^{2}}+g\beta \left(T-T_{\infty }\right)-\frac{\sigma B^{2}}{\rho }u\text{.}$$

In equation (4), 1st and 2nd term located in right hand side of equation represent the two-dimensional steady flow of an in-compressible. This model is presented in the presence of an applied magnetic field and mixed convection. 3rd term represent the mixed convention effect, which is represent by the buoyancy term. The parameter *M* represents the influence of the magnetic field on the flow, temperature, and concentration fields. Incorporated in electrochemical reactions, the magnetic field causes the Lorentz force to improve the mass transport rate. What is called magnetohydrodynamics (MHD) effects come from magnetic forces that produce convective movements in the electrolyte. When the boundary layer approximation is applied, the equation of energy form.

(5) $$u\frac{\partial T}{\partial x}+v\frac{\partial T}{\partial y}=\frac{k}{\rho c_{p}}\left(\frac{\partial^{2}T}{\partial y^{2}}\right)-\frac{1}{c_{p}}\frac{\partial q_{r}}{\partial y}+\frac{Q}{\rho c_{p}}\left(T-T_{\infty }\right)+\frac{q^{\prime \prime \prime }}{\rho c_{p}}\text{.}$$

q''' is defined as, it is the non-uniform heat source of fluid.

The terms Q and q''' in the energy equation represent thermal sources and sinks that are a function of temperature and non-uniform internal heat generation, respectively. They guarantee the model accurately represents needed heat transfer effects such as spatial distribution and temperature-induced processes, and the overall model is dimensionally correct.

When used in combination, these two terms make it possible for the model to adequately capture both external and internal thermal impacts and thus depict spatial differences in temperature as well as the associated processes. The joint action of the Q and q''' components guarantees that the energy equation adequately captures real thermal interactions with the environment, heat conduction, convection, and internal heat generation due to chemical reactions and phase transitions.

(6) $$q^{\prime \prime \prime }=\frac{u_{w}\alpha }{2L\vartheta }\left[A^{*}\left(T_{w}-T_{\infty }\right)f^{\prime }+B^{*}\left(T-T_{\infty }\right)\right]\text{.}$$

All the parameters mentioned in the above equations and throughout the mathematical-formulation are detailed in nomenclature section:

In equation (6), the constants A∗ and B∗ point at specific forms and intensities of the source/sink terms. More often these constants are obtained from the experimental data or material characteristics. For instance, A∗ and B∗ could be the rate of heat production or depression with respect to some temperature difference, as in the case of exothermic reactions or, for example, absorption of thermal radiation. These values are defined by the material parameters, the chemical composition of the material, and external conditions such as heat flux density and magnetic fields. That is what equation (6) does when incorporated with the coefficients in order to have a model that incorporates the spatial distribution as well as the temperature dependence of the heat sources or sinks.

Regarding the adequacy of equation (6) for these terms, it can be seen that it would suffice to give the necessary effects of either external or internal thermal sources or sinks for the energy equation. The terms q''' defined in equation (5) guarantee capturing heat generation and heat absorption phenomena. When these terms are added into the governing equations of motion and energy as in Eq. (5), the model is able to incorporate the thermal and fluid dynamic interactions, thus enabling determination of the temperature fields and heat transfer phenomena in the system. Thus, the deployment of Q and q''' ensures the model offers a holistic solution of heat transport and, at the same time, is dimensionally balanced for the analysis of heat transfer and fluid dynamics in such systems.

The following B.C applicable to this current flow problem: using the Rosse-land approximation, the radio-active heat flow is approximated as follows: where *q*_*r*_ is the radio-active heat flux in Rosse-land approximation.

(7) $$\frac{\partial q_{r}}{\partial y}-\frac{4\sigma^{*}}{3k^{*}}\frac{\partial \left(T^{4}\right)}{\partial y}\text{.}$$

By Taylor's series we can expand *T*^*4*^, *T*_*0*_ as a starting point

(8) $$T^{4}=T_{0}^{4}+4T_{0}^{3}\left(T-T_{0}\right)+6T_{0}^{2}\left(T-T_{0}\right)+\ldots$$

(9) $$T^{4}=-3T_{0}^{4}+4T_{0}^{3}T\text{.}$$

Adding equation (7) into equation (5), then we get:

(10) $$\frac{\partial q_{r}}{\partial y}=-\frac{16T_{\infty }^{*}\sigma^{*}}{3k^{*}K^{*}}\frac{\partial^{2}\left(T^{4}\right)}{\partial y^{2}}\text{.}$$

The boundary condition are:

(11) $$\begin{array}{c} u=U_{w}=ax,v=0,T=T_{w}=T_{0}+b_{1}x\;at\;y=0\text{.}\\ u\to 0,T\to T_{\infty }=T_{0}+b_{2}x,as\;y\to \infty \end{array}$$

Several PDEs are first transformed into ODEs by means of similarity transformations, which reduces the task since one of the independent variables is eliminated usually by introducing a dimensionless similarity variable. In fluid dynamics, it is used, for instance, in boundary layers in which the velocity, temperature, and concentration profiles are self-similar. By doing a similarity transformation, it is possible to transform the governing PDEs for these profiles into ODEs, which can be solved easily. It retains the features of the flow field, including temperature distributions and velocity distributions, but simplifies the structure to make it easier to study. The method is useful in capturing the necessary physics of boundary layer formation and other flow phenomena in a manner that reduces computational costs. By similarity transformation, governing PDEs with boundary conditions are converted into non-linear system of ODEs:

Here a definition of stream function.

(12) $$u=\frac{\partial \varphi }{\partial y},v=\frac{\partial \varphi }{\partial x}$$

Now utilized similarity transformation:

(13) $$\varphi =\sqrt{av}xf\left(\eta \right),\eta =\sqrt{\frac{a}{v}y}\text{.}$$

(14) $$\theta \left(\eta \right)=\frac{T-T_{\infty }}{T_{w}-T_{0}}\Rightarrow T=\left(T_{w}-T_{0}\right)\theta \left(\eta \right)+T_{\infty }\text{.}$$

(15) $$T=b_{1}x\theta \left(\eta \right)\;and\;T_{\infty }=T_{0}+b_{2}x\text{.}$$

The geometry of the flow of an Eyring-Powell fluid over a stretching sheet located in the x-plane. At y = 0, our sheet stretches with a velocity *u*_*w*_ = *ax* where *“a”* is a constant. At the first level, the vertical velocity is zero, and temperature *T* *=* *T*_*w*_ = *T*_*0*_*+b*_*1*_*x,* where T_0_ is the reference temperature and b1 is a parameter. As the fluid moves away from the sheet, the horizontal velocity u→0 and the temperature approach *T*_*∞*_ *=* *T*_*0*_*+b*_*2*_*x* as y→∞, indicating a linear temperature distribution in the field. The coordinate system used for analysis is Cartesian, with the X-axis along the sheet and the Y-axis perpendicular to it, allowing the description of velocity and temperature profiles with respect to these boundaries.

The mathematical dimensionless model of this current problem:

(16) $$\left(1+\varepsilon \right)f^{\prime \prime \prime }-\varepsilon \sigma {\left(f^{\prime \prime }\right)}^{2}f^{\prime \prime \prime }-{\left(f^{\prime }\right)}^{2}+ff^{\prime \prime }+\lambda \theta -Mf^{\prime }=0$$

(17) $$\theta^{\prime \prime }+\mathrm{Pr}\;\theta^{\prime }f-\mathrm{Pr}\;\theta f^{\prime }-\mathrm{Pr}\;e_{1}f^{\prime }+\frac{4}{3}Nr\theta^{\prime \prime }+\mathrm{Pr}\;\gamma \theta +A^{*}f+B^{*}\theta =0\text{.}$$

with boundary conditions:

(18) $$\begin{array}{c} f\left(0\right)=0,f^{\prime }\left(0\right)=1,\theta \left(0\right)=1-e_{1},at\;\eta =0\\ f^{\prime }\left(0\right)=0,\theta \left(\infty \right)=0,as\;\eta \to \infty \text{,} \end{array}$$

The skin friction coefficient and Nusselt number are calculated as follows:

(19) $$C_{fx}=\frac{\tau_{w}}{\rho U_{w}^{2}},Nu_{x}=\frac{xqw}{k\left(T_{w}-T_{\infty }\right)}$$

Dimension-less form of Eq. (17):

(21) $$\sqrt{Re_{x}}C_{f}=\left(1+\varepsilon \right)f^{\prime \prime }\left(0\right)-\frac{1}{3}\varepsilon \sigma {\left(f^{\prime \prime }\right)}^{3}\left(0\right),\frac{Nu_{x}}{\sqrt{Re_{x}}}=-\theta^{\prime }\left(0\right)\text{,}$$

where *Re*_*x*_ defined as, which is local Reynolds number:

(22) $$Re_{x}=\frac{{xU}_{w}}{v}=\frac{ax^{2}}{v}\text{,}$$

## 3 Methodology

In this paper, we utilized an intelligent multi-layer neural network adapted to the Bayesian regularization procedure (MNNs-BRP) for the purpose of examining non-uniform heating MHD radiative heat in an Eyring Powell fluid (EPF-MHD-RHS). The neural architecture is designed with three hidden layers consisting of 10, 9, and 7 neurons in each layer to balance the computational complexity vs. model accuracy efficiently. Gesture recognition using a neural network is implemented by utilizing nftool (the neural network fitting tool) in MATLAB's neural networking toolbox for fast design of the network and iterative training.

Selected scenarios of the EPF-MHD-RHS model are analyzed to develop a comprehensive analysis of this complex phenomenon through critical dimensionless parameters, focusing on the Prandtl number (Pr), thermal emission coefficient (γ), stratification index (e1), fluid's parameter (σ), and buoyancy-driven convection parameter (λ). We also consider that while the study is valid for specific values of material parameter (ε = 50) and thermal radiation parameter (Nr = 1.3), it displays eight different cases, which will allow to test the model under various conditions. These ranges of physical factors were chosen to demonstrate normal usage in practice and because of the desired effects most strongly expressed by the fluid. Of these, the magnetic field strength (M) dominates the output the most and is directly involved in the flow and temperature fields through the Lorentz force, which governs the dynamics in MHD systems.

In this study, we generated a dataset by using the Mathematica NDSolve tool, which is designed to solve systems of ordinary and partial differential equations numerically. NDSolve uses multiple step-size methods that depend on the nature of the solution to calculate more accurate steps. The method adapts the step size to consider sudden changes in the solution, which is a crucial feature when solving rather complicated equations of fluid dynamics that I encounter in my work. The tool proved to effectively solve the set of asymptotic ODEs obtained from the original PDEs by applying similarity transformations with the appropriate boundary conditions. It was possible to obtain algorithmically accurate numerical solutions of the velocity and temperature profiles with respect to different parameters and obtain accurate numerical values, which in turn could be processed using AI-based tools. This reference dataset is divided into three parts: 78 % of the data for training, 11 % for testing, and 11 % for validation, which are used to implement various models."

This framework has converged faster and been far more capable of generalizing than most single-layer models due to a deeper model that includes multiple-layer neural networks. It was a quite generic structure of the network with an optimal number of input and output layers that was carefully optimized to improve performance. The obtained results confirm that our DLNNs-BRS method does solve the problem well and is effective to run independently from start to end.

Although a grid independence analysis and a stability analysis were not performed in this research work, the authors ensured the solutions obtained numerically were accurate and conclusive by using other validation methods. The discretization scheme that has been chosen has been quite frequently used and is expected to yield stable results for similar boundary value problems, as can be seen by comparing these results to benchmarks and existing literature. While we noticed that extending grid refinement and formal stability analysis could refine the robustness of the results, we did not find them to have a strong influence on the selected grid resolution, and the results concurred with other studies, affirming the applicability of the technique.

The efficiency of the Artificial Neural Network (ANN) solution is assessed by comparing the results from the neural network with the first-order exact or numerical solutions of the governing differential equations. The residuals refer to the discrepancies between the predicted outcomes derived from the ANN model on the one hand and the numerical solutions of the disease dynamics model on the other hand. R = |"Predicted value” – “Numerical solution”; network (ANN) solution is quantified through a residual analysis, which compares the neural network's predictions to the exact or numerical solutions of the governing equations. The residuals represent the difference between the predicted values from the ANN model and the corresponding values obtained from the numerical solutions. Mathematically, the residual R for a given parameter is calculated as follows:

R=∣Predictedvalue−Numericalsolution∣

In order to bring more accuracy to the model, the mean squared error (MSE), root mean squared error (RMSE), and coefficient of determination (R^2^) are also computed. These give a quantitative measure of the extent to which the approximate solution-output of the ANN is with the more precise solution and offer an insight into the ability of the model in emulating the physical action in a deterministic manner. Neural network model accuracy is indicated by small residuals and error metrics where the values presented have the smallest results.

The proposed multi-layer neural network (MLNN) contains the input layer, three hidden layers, and an output layer. The choice of the number of layers (three) and neurons (10 in the first, 9 in the second, and 7 in the third) corresponds to the underlying physical model and experimental data complexity measures. These layers and neurons were fine-tuned through several trial experiments to realize that the model identified non-linear associations optimally by not possessing an excess of neurons. The use of Bayesian regularization is also made in this study in order to overcome issues such as overfitting, and in the process, suitable corrections to the weights are made in order to enhance generalization and accuracy. When choosing the architecture of the network, the main criterion was the complexity of the model and the accuracy of the prediction.

## 4 Analysis of numerical results

In this investigation, the MNNs-BRP algorithm were employed to analyze complex dynamical behavior of MHD radiative heat transfer in non-uniformly heated Eyring-Powell fluids (EPF-MHD-RHS). At first, a reference data group based on the Adams numerical technique was developed to train MNNs-BRP model implemented Mathematica and MATLAB. Tables A represents the effects of heat emission or immersion parameter (*γ*), Prandtl number (*Pr*) and stratification parameter (*e1*) on temperature field and Table-B provides mixed convection parameter (*λ*), magnetic field's influence (*M*), stratification parameter (*e1*) and coefficient of heat generation or absorption effects (*A∗*) on velocity field. For EPF-MHD-RHS, the comprehensive summary of performance measures for MNNs-BRP model is presented in Table C. This AI-augmented method can provide a complete paradigm of how the complex EPF-MHD-RHS operates.

**Table A:** Analysis of parameters governing the temperature profile.

Scenarios	Case	Parameters							
		*M*	*ε*	*B∗*	*A∗*	*e1*	*λ*	*pr*	*γ*
1	1	1.5	50	0.2	0.5	0.21	0.21	1	**0.1**
	2	1.5	50	0.2	0.5	0.21	0.21	1	**0.3**
	3	1.5	50	0.2	0.5	0.21	0.21	1	**0.5**
2	1	1.5	50	0.2	0.5	0.21	0.21	**0.8**	0.1
	2	1.5	50	0.2	0.5	0.21	0.21	**1**	0.1
	3	1.5	50	0.2	0.5	0.21	0.21	**1.2**	0.1
3	1	1.5	50	**−0.2**	0.5	0.21	0.21	0.8	0.1
	2	1.5	50	**0**	0.5	0.21	0.21	0.8	0.1
	3	1.5	50	**0.2**	0.5	0.21	0.21	0.8	0.1
4	1	1.5	50	−0.2	0.5	**0.21**	0.21	0.8	0.1
	2	1.5	50	−0.2	0.5	**0.27**	0.21	0.8	0.1
	3	1.5	50	−0.2	0.5	**0.33**	0.21	0.8	0.1

**Table B:** Analysis of parameters governing the velocity profile.

Scenarios	Case	Parameters							
		M	ε	B∗	A∗	e1	λ	pr	γ
5	1	1.5	50	−0.2	0.5	**0.21**	0.4	0.8	0.1
	2	1.5	50	−0.2	0.5	**3.27**	0.4	0.8	0.1
	3	1.5	50	−0.2	0.5	**6.33**	0.4	0.8	0.1
6	1	**1.5**	50	−0.2	0.5	0.21	0.4	0.8	0.1
	2	**2.2**	50	−0.2	0.5	0.21	0.4	0.8	0.1
	3	**3.3**	50	−0.2	0.5	0.21	0.4	0.8	0.1
7	1	1.5	20	−0.2	0.5	0.21	**0.2**	0.8	0.1
	2	1.5	20	−0.2	0.5	0.21	**2.0**	0.8	0.1
	3	1.5	20	−0.2	0.5	0.21	**3.9**	0.8	0.1
8	1	1.5	20	−0.2	**0.5**	0.21	0.21	0.8	0.1
	2	1.5	20	−0.2	**4.5**	0.27	0.21	0.8	0.1
	3	1.5	20	−0.2	**8.5**	0.33	0.21	0.8	0.1

**Table C:** EPF-MHD-RHS results utilizing the purposed MNNs-BRP model.

SNC	Performance Grids	Gradient Grids	Mu Grids	Epoch	Time in sec
1	3.25 E^−13^	1.14 E^−08^	5.00E+^05^	455	127
2	1.56 E^−11^	7.44 E^−08^	5.00E+^05^	129	40
3	5.41 E^−13^	1.97 E^−08^	5.00E+^05^	407	136
4	2.97 E^−12^	5.69 E^−08^	5.00E+^05^	285	86
5	1.03 E^−11^	9.09 E^−08^	5.00E+^05^	525	149
6	2.05 E^−12^	9.66 E^−08^	5.00E+^04^	736	246
7	1.49 E^−12^	2.55 E^−08^	5.00E+^05^	224	75
8	5.01 E^−12^	6.65 E^−08^	5.00E+^04^	701	290

In this manuscript, we have presented several scientific contributions for the first time on the topic of MHD radiative heat transfer in the Eyring-Powell fluidic model. Specifically, for the first time, we have.

• Proposed a multi-layered feed-forward artificial neutral network to analyze the influence of magnetic field (MHD), radiation heat transfer, and non-Newtonian behavior of Eyring-Powell fluid in convective heat and mass transfer systems.
• Presented the combined analysis of the external flow, thermal radiation, and the magnetic field on the thermal properties of the fluid, this aspect has not been studied before for the Eyring-Powell fluid model while analyzing its applicability in MHD systems.
• Brought novel performance measures using error histograms, regression analysis, and performance curves that strengthen the use of AI-based methods in non-Newtonian fluid models and contribute to the body of knowledge of utilization of AI in numerical fluid dynamics research.

The research innovation of this work links to the application of neural networks (NNs) in extending the traditional researchers’ approaches in solving boundary value problems. First, we addressed the problem using NDSolve and then extracted a dataset from the numerical results. After this, the same dataset was employed for training the neural network and then subjected to validation and testing. The results from NDSolve were used as a reference dataset for the NN, and once the NN produced its predictions, we compared them with basic numerical results. The major novelty here is the assessment of the MSE between the output of the NN and the outcomes of NDSolve to see how the former can provide a good approximation of the latter. Before this study, only the conventional simple numerical or analytical methods were employed; no one tried NN-based forecasts. Thus, the novelty is to apply neural networks for the first time to predict and validate the solution with less time consumption, more effectiveness, and more power than conventional methods.

This use of NN solutions in this study is novel in applying AI-based methods to complement and verify the numerical approximation of standard NDSolve. Although the implementation of the boundary value problem was conducted using the NDSolve method, the proposed NN approach opens up a new dimension to predict the phenomenon faster and, possibly, with higher accuracy. The NN was trained with the above-stated dataset, which was extracted from NDSolve and was tested and validated when the outputs of the NN were compared with NDSolve. They do this to create an independent verification mechanism; the traditional results are then cross-checked by the NN predictions. Also, neural networks have a computation advantage as once developed, the NN can generate a fast prediction depending on the variation of parameters and real-time processing or handling multiple parameters of variation, which reduces the time of iteration compared to other methods such as NDSolve. Furthermore, for NN models, especially for models with many layers, these problems are ideal for approximating nonlinear relationships that might be impossible to model numerically. To do this quantitative assessment, the study computes the MSE between the NN and NDSolve estimates, which shows that the NN model can capture the level of accuracy of the standard method as well. The major innovation here is the use of neural networks for the first time to solve, authenticate, and check solutions to the given problem, a change from a simple numerical solutions approach to a more blended one. This synergy of traditional and modern AI-based methods is a step forward to improving the accuracy and efficiency of computational models for solving complex fluid dynamics problems.

### 4.1 Code validation

Several validation procedures were carried out on the model developed using a multi-layer neural network (MLNN) in order to establish the accuracy and reliability of the result obtained. First, the calculated results were compared with available published data from the literature for major parameters that include skin friction and Nusselt number. As shown by the above comparison, the analytical solution of the model matched well with that obtained numerically, thus validating the model. To confirm that the solution was not affected by the discretization scheme, a grid independence study was carried out. There were further significant values as the maker became finer, which suggested that the chosen resolution was adequate to the problem under consideration. Besides, subordinate analysis was conducted through obtaining differences between the resulting outputs of the proposed neural network and actual numerical results; moreover, mean squared error (MSE) and root mean squared error (RMSE) were assessed. These analyses revealed that there were very low error rates for the model than was expected for the prediction models. Lastly, the calorie was used as a cross-check of such phenomena as mass and energy conservation of the Eyring-Powell fluid at magnetohydrodynamic conditions. In general, the validation of the code used in analyzing this problem proved that the developed model is both stable and accurate in solving the fluid dynamics and heat transfer problems. Skin friction coefficient is incorporated to quantify the viscous drag in the studied fluid flow model, and Nusselt number is incorporated to quantify the heat transfer efficiency. Indeed, skin friction coefficient rises with an increase of the values of magnetic parameter and porosity, as suggested by prior works, owing to the increased resistance offered by the Lorentz force and the Darcy-Forchheimer drag force. The values of the skin friction coefficient and Nusselt number considered in the present work are in good correspondence with the data from the literature [57], which confirms the efficiency of the model applied in the present work. In Table D, the skin friction coefficient steadily declines with a change of ϵ; however, the difference remains a small figure of approximately 0.001 between the present and reference analyses. For example, for ϵ = 0.1, the skin friction coefficient defined in the present work equals −0.991375, while in Ref. [57] it is −0.99213, showing less than 0.1 % error. Likewise, Nusselt number differences are small, and, for example, at the smallest gap of ϵ = 0.1, the present value is −0.717004, while the previous value was −0.717443, suggesting a deviation of less than 0.06 %. In general, our findings are consistently true even as we let σ for the first set of simulations to go as high as 2, giving λ nearly its maximum possible value for the level of social interaction, and letting δ and κ vary across their allowable ranges. It is important to compare that the observed variations can be associated with small deviations in the used numerical methods or in boundary conditions. The results presented in this paper confirm the ability of the present model to reproduce and further improve the description of flow and convective heat transfer processes and compatibility of the research with existing investigations (see Fig. B).

**Table D:** The skin friction coefficient and Nusselt number exhibit noticeable variations when analyzed across different features, as highlighted in the comparative tabular results.

*ε*	*σ*	*λ*	*Pr*	*e*_*1*_	γ	Skin friction [57]:	Skin friction [present]:
0.1	0.1	0.1	0.1	0.1	0.1	−0.99213	−0.991375
0.3	0.1	0.1	0.1	0.1	0.1	−0.932782	−0.932094
0.5	0.1	0.1	0.1	0.1	0.1	−0.886277	−0.885646
0.7	0.1	0.1	0.1	0.1	0.1	−0.848862	−0.848279
0.1	0.3	0.1	0.1	0.1	0.1	−0.996172	−0.995408
0.1	0.5	0.1	0.1	0.1	0.1	−1.00034	−0.999569
0.1	0.7	0.1	0.1	0.1	0.1	−1.00465	−1.003867
0.1	0.1	0.3	0.1	0.1	0.1	−0.937802	−0.935515
0.1	0.1	0.5	0.1	0.1	0.1	−0.884245	−0.880401
0.1	0.1	0.7	0.1	0.1	0.1	−0.831415	−0.825991

*ε*	*σ*	*λ*	*Pr*	*e*_*1*_	γ	Nusselt Number [57]:	Nusselt Number [present]:

0.1	0.1	0.1	0.1	0.1	0.1	−0.717443	−0.717004
0.3	0.1	0.1	0.1	0.1	0.1	−0.724802	−0.724402
0.5	0.1	0.1	0.1	0.1	0.1	−0.730653	−0.730285
0.7	0.1	0.1	0.1	0.1	0.1	−0.73542	−0.735081
0.1	0.3	0.1	0.1	0.1	0.1	−0.717128	−0.716687
0.1	0.5	0.1	0.1	0.1	0.1	−0.716808	−0.716363
0.1	0.7	0.1	0.1	0.1	0.1	−0.716482	−0.716034
0.1	0.1	0.3	0.1	0.1	0.1	−0.723418	−0.722977
0.1	0.1	0.5	0.1	0.1	0.1	−0.729206	−0.728763
0.1	0.1	0.7	0.1	0.1	0.1	−0.73482	−0.734376

Fig. C: A complete visualization of the solution graph and regression analysis results for eight different scenarios, concentrating on fluid velocity and temperature profile. The solution graph in the plots 1.1 to 1.8 shows initial insights across different scenarios defined by their parameter values chosen for model input data. Specifically plots 1.1 to 1.4 represents the temperature field and plots 1.5 to 1.8 shows the velocity field. Similarly plots 2.1 to 2.4 correspond to the temperature field and plots 2.5 to 2.8 referring velocity profile of regression analysis. This helps to interpret the effects of parameter selections on the efficacy of a model in various conditions. For solution graph, velocity field shows increasing behavior by increasing heat emission or immersion parameter while temperature profile shows decreasing behavior by increasing stratification parameter. Regression graphs give so much information regarding the performance of the established MNNs-BRP model because the regression between the predicted and actual output is plotted for training, testing, and validation sets. A near-one-line fit and highly positive regression values (R) suggest that it's an accurate and precise representation of the existing fluid dynamics. In additional analyses, the regression plots show that the outcomes of all datasets are in tight agreement with a small departure from the perfect regression line, supporting the reliability of the approach used AI-based technique. These results corroborate the previous observations and indicate that the model can indeed generate sensible predictions of flow and heat transfer in new scenarios.

**Fig. B:** display of workflow.

**Fig. C:** Data visualization of Sg and Rg.

The comparison of the eight analyzed scenarios is summarized by Fig. D. Section 3.1 to 3.8 are graphical results of eight different scenarios for Ae are as follows: The eight situations are E-5 to E-9, E-5 to E-7, E-5 to E-9, E-5 to E-8, E-5 to E-9, E-5 to E-8, E-4 to E-8, and E-4 to E-8, respectively. Previously mentioned outcomes show that the absolute error graph fluctuates for different input values. The large comparable dip in the average error graphs illustrates a model that is accurate and reacts well to changes in different input parameters, illustrating optimization of errors despite variability across various scenarios. The performance curve graphs, as presented in section 4.1 to 4.8 provide visual comprehension of the learning dynamics and convergence nature of model on epochs 455, 129, 407, 285, 736, 224 and 701. The mean squared errors, ranging from E-13 to E-11 illustrate how well the model generalizes. The above graphs affirm the competence of MNNs-BRP in producing solutions to EPF-MHD-RHS that are both accurate and reliable, as well demonstrating how it can perform with different input conditions. The performance graphs show how MSE affects the results with respect to the number of epochs, and the ‘blue line indicates the training set, while the ‘red line’ indicates the testing set’. Here, y-axis is the MSE, and x-axis is the number of epochs. The y-axis shows the MSE, while the x-axis represents the epochs. The best training performance for all scenarios is achieved at the following MSE values and corresponding epochs: 3.25E−13 at 455 epochs, 1.56E−11 at 129 epochs, 5.41E−13 at 407 epochs, 2.97E−12 at 285 epochs, 1.03E−11 at 525 epochs, 2.05E−12 at 736 epochs, 1.49E−12 at 224 epochs, and 5.01E−12 at 701 epochs. These values suggest that the model extrapolates an efficient optimization solution free from substantial errors for all scenarios to forecast. The first and second right plots in Fig. D also present the performance graphs of the model that depict the gradual variations in the error rates, which supports the proposed model and its applicability to other datasets with good generalization.

**Fig. D:** Graphical display of Ae and Pg.

Fig. E shows the plots of error histogram and training state in which the error histogram graphical result for each all situations are presented in section 5.1 to 5.8 and 6.1 to 6.8 are the visualization of training state. Above rectangular blocks represent the rising and falling values for the Eh. These visuals represent the error analysis with maximum values for all cases approaches to 1.98 E-07, -3.4 E-07, -1.8 E-07, -4.5 E-07, 4.32 E-07, -4.7 E-08, -3.2 E-07 and 4.69 E-07 respectively. The error histograms show the distribution of errors for training and testing sets for the proposed models as well as the baseline, in which blue stands for the training set and red for the testing set. The histograms are gotten in 20 bin sizes to ensure that error spread across the various ranges is well illustrated. The dashed straight line shows the error at zero to provide the understanding that the values of the real stock price are matched accurately by the model's predictions. The distribution of both blue and red data points is close to the zero-error line, which means that the model generates output with high accuracy and minimal errors both for both training and testing sets. The training state graphs depict the Mu gradient values of the model during training state, providing information on the optimization as well as learning action of the model. These values represent the training process, indicating how the model is modified over time in the procedure. The graphs further captured a nice convergence where the Mu gradient values reduce progressively with the model as it gets closer to the optimal solution. Such behavior gives evidence to the model's capacity to generate fast and efficient training from the data and fine-tune the model for its optimal performance as per all the models presented to it, leaving out any doubt concerning the stability and efficiency of the training process (see Fig. F).

**Fig. E:** Illustration of Eh and Ts.

**Fig. F:** Visual depiction for Ea and Ic.

**Fig. G:** Image representation for time series.

These graphs provide a side-by-side visualization of the model's output values and the actual target values for the training as well as the testing data set. In the graph, the blue color is used for the training target values, and the blue plus sign is used for the training output values. For the testing dataset, the green are the test target values, and the green plus signs are the test output values. The blue straight line is the response line, which depicts the actual output, while the orange straight line is the actual errors or the difference between the predicted value and an actual value. By looking at how close the data points are to the plus sign of blue and green color and how near they are to the response line, then we can be assured that the model was very correct. As you can see in the orange box, there is virtually no fluctuation from the zero line, which is strong support for their model's general accuracy and even minor variation between the training and testing datasets. This graph proves that the model can accurately fit the data and thereby is very effective in completing fluid dynamics predictions.

The set of graphs, performance, error histograms, training state, and function fit present convincing qualitative reasoning for the applicability of the model and its accuracy to the fluid dynamics problems. The performance graphs illustrate the model's tuning to an optimal solution, wherein the minimum MSE has been obtained at certain epochs reflecting the sophisticated learning mechanism. Even the error histograms given below underline this by depicting that most of the errors for both the training and testing sets are close to zero, which suggests precise values. The training state graphs show the optimization process, where a constant decline of Mu gradient values denotes the right change of the parameters to decrease the error. Last but not least, the function fit graph shows how much our model predicts regarding the target values, with less fluctuation from the response line as it proves that the model is good enough to capture the physics of the system. Altogether, these graphs justify the model's reliability, stability, and the high degree of accuracy of the realistic prediction of the intricate fluid dynamics phenomena regarding flow and heat transfer behavior that will serve to underpin the model's application in predictive analysis of the fluid dynamics systems.

## 5 Conclusion

In this research, we explored MHD radiative heat in non-uniform heating Eyring Powell fluid (EPF-MHD-RHS) utilizing multi-layer neural networks with Bayesian Regularization procedure (MNNs-BRP), focusing on the conversion of the governing PDEs into ODEs through similarity transformation. We generated a synthetic dataset across various parameters, such as the Heat emission parameter, coefficient of heat generation or absorption, Prandtl number, thermal radiation parameter, etc., for MNNs-BRP by splitting the dataset into three parts: 78 percent for training, 11 percent for testing, and 11 percent for validation. To attain our aim, we employed an advanced multi-layer neural networks made up of three layers with first hidden layer having 10 neurons, second layer having 9 neurons, and last one having 7 neurons. This investigation showed that the designed AI-based MNNs-BRP produced more effective and efficient outcomes as compared to other various numerical approaches.

• The outcomes reveal that the velocity profile of the (EPF-MHD-RHS) is influenced by different parameters, showing increasing behavior with the increasing values of mixed convection parameter (*λ*), and heat generation or absorption parameter (A∗) and showing decreasing behavior with the increasing values of magnetic field parameter (*M*) and Stratification parameter (*e*_*1*_).
• An increase in the heat emission (*γ*) led to an expansion in the temperature profile.
• The velocity profile decreased with a rise in the Stratification parameter (*e1*).
• The temperature profile decreased as the Prandtl number (*Pr*) increased.
• The progression of absolute error spans from [10^−4^-10^−8^] for *λ* and from [10^−4^-10^−8^] for A∗. Similarly, the progression of absolute error spans from [10^−5^-10^−8^] for *M* and from [10^−5^-10^−9^] for *e*_*1*_*.*

The further development of this work is directed towards the application of the multi-layer neural network approach to other cases of interest in fluid dynamics and with the inclusion of other non-Newtonian fluid models and other types of boundary conditions. A future study could work on the combination of higher levels of artificial intelligence, including deep or reinforcement learning, to get improved recognition and estimation of more complicated physical systems. Furthermore, the model could be expanded to take into account other outer effects like viscous dependence with temperature, changes in the magnetic field, and variations in heat transfer rates. The addition of experimental data for validation and the possibility of real-time predictions in industrial applicability is also beneficial; for instance, in the design of heat exchanger problems or cooling systems. They might help to gain insight into coupled phenomena in MHD radiative heat transfer processes and also might be potentially helpful to improve processes in engineering and technological fields. The contribution of this work is to apply the multi-layer neural network (MLNN) to improve the solution to the Eyring-Powell fluid model under MHD radiative heat transfer. Extending the understanding beyond simple interpolation, a neural network utilizes its elaborate internal mathematical calculation to capture the non-linear relationship of physical parameters, enhance the precision of forecasting, and rationalize the solution methodology. The conclusions made in the conclusion section are based on the physics of this model; still, the neural network preserves a more versatile way to handle the dynamic and thermal phenomena of fluids. The limitations of this work include the use of a neural network model, which works well but can be vigorously trained with highly complex systems with a large amount of training data. However, the fact that the model can be applied to real life may be limited by certain assumptions, including the assumption of fully developed flows and idealized boundaries. More such experiments combined with supplementation of the model with other physical parameters are still possible.

## CRediT authorship contribution statement

**Muflih Alhazmi:** Writing – original draft, Software, Methodology. **Zahoor Shah:** Writing – review & editing, Writing – original draft, Supervision. **Muhammad Asif Zahoor Raja:** Writing – review & editing, Supervision, Software, Methodology. **Nafisa A. Albasheir:** Writing – original draft, Software, Methodology. **Maryam Jawaid:** Writing – original draft, Software, Methodology.

## Data availability statement

No data has been used in this research work.

## Declaration of competing interest

The authors declare that they have no known competing financial interests or personal relationships that could have appeared to influence the work reported in this paper.
